The article "Analysis of Systolic Blood Pressure Level and Short-Term Variability in Masked Hypertension" was retracted in 2023. Reasons: signs of a paper mill; suspected computer-generated content; unreliable results or conclusions; concerns about the data.

# Analysis of Systolic Blood Pressure Level and Short-Term Variability in Masked Hypertension

**DOI:** 10.1155/2022/8016893

**Published:** 2022-04-09

**Authors:** Yinjing Hou, Bo Liu

**Affiliations:** Department of Geriatrics, Beijing Tongren Hospital, Capital Medical University, Beijing 100730, China

## Abstract

**Background:**

Patients with masked hypertension are at an elevated risk of cardiovascular events and all-cause death. This risk is close to that of sustained hypertension. The mean value and short-term variability of systolic blood pressure are considered to be risk factors for organ damage in hypertension.

**Objective:**

To investigate the mean value and short-term variability of systolic blood pressure in patients with masked hypertension.

**Methods:**

According to the results of in-clinic and ambulatory blood pressure measurement, participants were divided into four groups: normotension group, controlled hypertension group, masked hypertension group, and sustained hypertension group. The mean value and short-term variability of systolic blood pressure of masked hypertension group were evaluated by comparison with the other three groups.

**Results:**

A total of 250 subjects were enrolled, with an average age of 65.46 ± 8.76 years, and 166 (66.4%) were male, including 62 in the normotension group, 78 in the controlled hypertension group, 69 in the masked hypertension group, and 41 in the sustained hypertension group. Compared with the normotension group and controlled hypertension group, the mean value, blood pressure load, standard deviation, and coefficient of variation of systolic blood pressure over 24 hours and during the day and night, were all higher in the masked hypertension group (*P* < 0.05), while the rate of the nocturnal systolic blood pressure decline was lower (*P* < 0.05). There were no statistically significant differences in the above indexes between the masked hypertension group and sustained hypertension group (*P* > 0.05).

**Conclusion:**

There are higher mean value of systolic blood pressure and greater short-term variability in masked hypertension patients. Identification of masked hypertension is an important challenge in the clinic.

## 1. Introduction

Masked hypertension (MH) has recently been identified as a unique hypertension phenotype that occurs in both treated and untreated patients. MH is characterized by an elevated blood pressure when the patient is out of the clinic but a normal blood pressure when the patient is in the clinic. MH accounts for at least 15% of people with apparently normal blood pressure in the clinic [1, 2], but reports suggest that this figure may be an underestimate of its prevalence. Because MH patients can be in a state of elevated blood pressure for long periods of time, the clinical outcomes tend to be different from patients with true normotension. In particular, mounting evidence suggests that MH leads to increased risks of organ damages that are similar to those associated with sustained hypertension (SH) [2–4].

The article "Analysis of Systolic Blood Pressure Level and Short-Term Variability in Masked Hypertension" was retracted in 2023. Reasons: signs of a paper mill; suspected computer-generated content; unreliable results or conclusions; concerns about the data.

Although the harm of MH has been well recognized, limited research studies on the characteristics of systolic blood pressure (SBP) are available. Notably, multiple studies have shown that the elevated SBP impacts the risks of all-cause mortality, heart failure, stroke, and end-stage renal disease more than diastolic blood pressure does [5–7]. Accordingly, SBP tends to be the key target of blood pressure management in official guidelines [1, 2]. The level and variability of SBP are closely related to the progress of arteriosclerosis, which are the main predictive factors in predicting cardiovascular events and all-cause death [5]. Therefore, both the level of SBP and its variability may represent important factors affecting the prognosis of MH.

There are a few studies analyzing the differences of blood pressure variability among different phenotypes of hypertension [8, 9]. However, few studies have focused on the characteristics of SBP in patients with MH. The purpose of this study is to discuss the reasons for higher target organ damage of MH reported in the past by describing the differences in the average value and short-term variability of SBP over 24 hours and during the day and night among patients with normotension, controlled hypertension, MH, and SH.

## 2. Materials and Methods

### 2.1. Study Participants

A cross-sectional study was performed. Information was collected from patients hospitalized in Beijing Tongren Hospital whose vitals were stable from July 2020 to July 2021. This study was approved by Beijing Tongren Hospital Ethics Committee (no. TRECKY2021-192).

### 2.2. Inclusion and Exclusion Criteria

Details on the inclusion and exclusion of participants are shown in Figure 1. The inclusion criteria were as follows: age ≥45 years old, agreed to participate in the trial, and signed the informed consent form. The diagnostic criteria for hypertension were in line with the 2018 European Society of Cardiology/European Society of Hypertension（ESC/ESH）Guidelines for the Management of Arterial Hypertension [1] (hereinafter referred to as guidelines). The exclusion criteria were as follows: (1) diagnosis of SH; (2) glycosylated hemoglobin HbA1c >7.5%; (3) left ventricular ejection fraction ≤50%; (4) previous diagnosis of myocardial infarction and performing percutaneous intervention or coronary artery bypass grafting; (5) heart failure; (6) cerebrovascular disease, including stroke or transient ischemic attack; (7) carotid or cerebral artery revascularization; (8) hyperthyroidism (TSH <0.1 mU/L) or hypothyroidism (TSH >10 mU/L); (9) liver diseases (jaundice hepatitis, or cirrhosis, or liver failure); (10) chronic kidney disease 4 or above (eGFR <30 mL/min/1.73 m^2^); (11) severe infectious diseases or autoimmune diseases; and (12) malignant tumors; mental disorders. Participants were constantly enrolled in the study. A total of 250 participants were eligible. All participants were collected a completed medical history survey and underwent laboratory examination and ambulatory blood pressure monitoring.

The article "Analysis of Systolic Blood Pressure Level and Short-Term Variability in Masked Hypertension" was retracted in 2023. Reasons: signs of a paper mill; suspected computer-generated content; unreliable results or conclusions; concerns about the data.

### 2.3. Data Collection

#### 2.3.1. Epidemiological Questionnaire

A questionnaire was completed by participants and then verified by the study physician. The questionnaire items included demographic information, educational background, lifestyle (such as physical activities and use of alcohol or tobacco), types of antihypertension drugs and years medications were used, other complications, and family history. The use of alcohol was defined as having consumed alcohol more than 12 times in the past 12 months [10]. Physical activities were defined as at least 150–300 minutes of moderate-intensity aerobic activity per week; or at least 75–150 minutes of high-intensity aerobic activity [11].

#### 2.3.2. Anthropometric and Biochemical Measurements

Standard instruments were used for all measurements. Anthropometry included height, weight, body mass index (BMI), and blood pressure. Biochemical tests included fasting blood glucose (FBG), HbA1c, triglycerides (TG), total cholesterol (TC), high-density lipoprotein cholesterol (HDL-C), and low-density lipoprotein cholesterol (LDL-C). The morning after an overnight fast, blood samples were collected from the forearm vein into vacuum tubes containing EDTA. FBG was measured by the hexokinase method. Determination of cholesterol and triglycerides were performed by enzymatic methods using commercially available kits (Beijing Tongren Hospital Clinical Laboratory).

#### 2.3.3. In-Clinic Blood Pressure Measurements

Participants were instructed to rest in the sitting position for at least 5 minutes prior to measurements. Blood pressure was measured on the same arm throughout the study with a Hem-7051 blood pressure monitor (Omron, Kyoto, Japan). For each measurement, three consecutive blood pressure readings were obtained, and the average of these blood pressure readings was submitted to the clinic.

#### 2.3.4. Twenty-Four-Hour Ambulatory Blood Pressure Monitoring

An ambulatory blood pressure monitor (Vasomedical BIOX Ambulatory Blood Pressure Monitor) was installed on the passive arm of each participant to automatically measure and record blood pressure. In the daytime, it was programmed to perform measurements every 20 minutes between 08:00 and 22:00. In the nighttime, it was programmed to perform measurements every 60 minutes after 22:00. Participants wore the ambulatory blood pressure monitor for 24 hours. If a record contained 70% of the programmed readings, the coverage time was greater than 20 hours and there were at least 20 readings during the day and at least 7 readings during the night, the record was considered effective [2]. Blood pressure values were weighted over the time interval between successive readings.

The article "Analysis of Systolic Blood Pressure Level and Short-Term Variability in Masked Hypertension" was retracted in 2023. Reasons: signs of a paper mill; suspected computer-generated content; unreliable results or conclusions; concerns about the data.

### 2.4. Grouping

The participants were divided into four groups according to in-clinic and ambulatory blood pressure values as guided by guidelines [1]. The four groups were assigned as follows. Group 1 was the normotension group: there was no history of hypertension, the blood pressure in the clinic was less than 140/90 mmHg, and the ambulatory blood pressure parameters were not within the range of hypertension. Group 2 was the controlled hypertension group: there was a history of hypertension, the blood pressure in the clinic was less than 140/90 mmHg, and the ambulatory blood pressure parameters were not within the range of hypertension. Group 3 was the MH group: the blood pressure in the clinic was less than 140/90 mmHg, and the ambulatory blood pressure parameters were within the range of hypertension. Group 4 was the SH group: the blood pressure in the clinic was greater than 140/90 mmHg, and the ambulatory blood pressure parameters were within the range of hypertension. Specifically, for ambulatory blood pressure parameters to be within the range of hypertension, the 24-hour average blood pressure was at least 130/80 mmHg, or the daytime average blood pressure was at least 135/85 mmHg, or the nighttime average blood pressure was at least 120/70 mmHg.

### 2.5. Statistical Analysis

The data were recorded by two people and consistency test was carried out. EpiData 3.1 was used to input data. The SPSS 22.0 statistical software was used to process descriptive statistics and difference analyses. Counting data were described by frequency distributions and were analyzed by chi-square tests. After a Kolmogorov–Smirnov normality test, the measurement data conforming to a normal distribution were expressed as‾*X* ± SD, and the analysis of variance was used. The data that did not conform to a normal distribution were represented by the *M* (*Q*1, *Q*2) and were analyzed by the Mann–Whitney *U* test and the Kruskal–Wallis test. All factors were subjected to bilateral tests. Differences for which *P* < 0.05 were considered to be statistically significant.

The article "Analysis of Systolic Blood Pressure Level and Short-Term Variability in Masked Hypertension" was retracted in 2023. Reasons: signs of a paper mill; suspected computer-generated content; unreliable results or conclusions; concerns about the data.

## 3. Results

A total of 250 participants were included in this cross-sectional study. The average age of participants was 65.46 years, and 166 (66.4%) of the participants were male. The normotension group included 62 cases, the controlled hypertension group included 78 cases, the MH group included 69 cases, and the SH group included 41 cases. There were statistically significant differences in age, gender, BMI course of hypertension, number of antihypertension drugs, status of diabetes, and hyperlipidemia as well as levels of TG, FBG, and HbA1c among the four groups (Table 1).

The SBP parameters of ambulatory blood pressure monitoring among four groups are summarized in Figure 2. The average value, the standard deviation, and the coefficient of variation of SBP in all three time frames (24 hours, daytime, and nighttime) were significantly higher in the MH group compared with both the normotension group and the controlled hypertension group. The blood pressure load over all three time frames was also significantly higher in the MH group compared with both the normotension group and the controlled hypertension group (*P* < 0.05). The rate of the nocturnal SBP decline was lower in the MH group compared with both the normotension group and the controlled hypertension group. The above indexes regarding SBP in the MH group were not statistically different from those in the SH group (*P* > 0.05).

## 4. Discussion

In this study, we found that, as compared with participants with normal blood pressure or controlled hypertension, those with MH had a higher average value and blood pressure load and a higher standard deviation and coefficient of variation of SBP over all tested time frames. The rate of the nocturnal SBP decline was lower in participants with MH. These results suggest that the level of SBP and its short-term variability during all time periods (including night) are higher in patients with MH than in those with normal blood pressure. These differences support the idea that the blood pressure of people with MH, are in fact different from those of people with truly normal blood pressure. In addition, these differences in blood pressure suggest that their prognosis must be different. Therefore, it is important that we should pay much attention to identifying patients with MH.

In this study, we found that MH patients had generally a high SBP level, which would be expected to negatively impact blood vessels and to result in subsequent damage to multiple organs. High SBP has also been associated with the progression of arteriosclerosis. For example, in a meta-analysis, after adjusting for demographic indicators, a correlation was found between SBP and arteriosclerosis progression. Specifically, after adjusting for age, patients' pulse wave velocity was shown to increase by 1.14 m/s for every 20 mmHg increase in SBP. However, the correlation between mean arterial pressure or diastolic pressure and pulse wave velocity was weak [5]. Arteriosclerosis plays a key role in hypertension-related clinical outcomes and is a powerful predictor of cardiovascular events and all-cause death [12, 13]. Therefore, current hypertension guidelines identify arteriosclerosis as one of the markers of target organ damage. Similarly, these guidelines commonly advise to reduce arteriosclerosis by drastically lowering blood pressure, mainly SBP, to reduce the occurrence of serious organ damage [1, 2]. An important outcome of this study was that SBP tended to be high in patients with MH both during the daytime and nighttime, and the rate of the nocturnal SBP decline was low. These factors are bound to affect the prognosis of MH patients. Studies have shown that high nighttime blood pressure is more closely associated with risks of cardiovascular events and all-cause death than daytime blood pressure [14–16]. Both lifestyle factors, including work stress and lack of sleep, and biological factors, including metabolic syndrome and sleep apnea syndrome, are MH risk factors that all enhance the activities of nocturnal autonomic nerve, resulting in the increase of nighttime SBP. Therefore, controlling nighttime SBP, via the mitigation of risk factors and the appropriate timing of drug administration, will become one of the keys of MH management in the future.

The article "Analysis of Systolic Blood Pressure Level and Short-Term Variability in Masked Hypertension" was retracted in 2023. Reasons: signs of a paper mill; suspected computer-generated content; unreliable results or conclusions; concerns about the data.

We also found that MH patients have high SBP variability, which also helped to explain the previously reported high cardiovascular risks in MH patients. Multiple studies have demonstrated the links between SBP variability and risks of coronary heart disease, stroke, end-stage renal disease, and all-cause death that are stronger than SBP itself [17–19]. The blood pressure variability may be affected by both sympathetic regulation and arterial elasticity. The results of this study showed that the variabilities of SBP in the MH group and the SH group were similar, which were consistent with the results of previous studies [8]. It may be explained by a similar disturbance of the regulation of sympathetic function. Siddiqui et al. [17] compared the sympathetic nerve activities of patients with controlled hypertension and those with masked uncontrolled hypertension (MUCH) both in the clinic and out of the clinic. They found that blood pressure variability, urinary catecholamine, and urinary norepinephrine levels out of the clinic were significantly higher in patients with MUCH than those with controlled hypertension. It was therefore speculated that the enhancement of sympathetic nerve activities out of the clinic promoted the development of MUCH. Another study found that sympathetic nerve activities in patients with MH was significantly higher than those with normal blood pressure [20]. These studies showed abnormal sympathetic activities in MH patients that resulted in higher blood pressure variability as compared to patients with normal blood pressure.

The article "Analysis of Systolic Blood Pressure Level and Short-Term Variability in Masked Hypertension" was retracted in 2023. Reasons: signs of a paper mill; suspected computer-generated content; unreliable results or conclusions; concerns about the data.

On the other hand, although the effect of arteriosclerosis on blood pressure variability is not fully understood, the possibility of an alternate direction of causation cannot be ruled out. A major determinant of blood pressure variability depends on baroreceptor sensitivity [21]. When the vascular structure changes significantly, it may reduce the sensitivity of arterial baroreceptors by limiting the extension of baroreceptors, and the lower sensitivity would be expected to lead to increased blood pressure variability [22, 23]. Moreover, atherosclerosis itself may enhance blood pressure fluctuations associated with small changes in cardiac output. Notably, the inverse relationship between blood pressure variability and baroreceptor sensitivity has not been confirmed by prospective studies. However, no matter the reason, the increase of blood pressure variability in MH patients may cause vascular endothelial dysfunction or injury, promote inflammatory responses and immune activation, and lead to atherosclerosis, ischemic myocardial injury, or damage to target organs [24].

## 5. Limitations

This study had several limitations. First, the sample size of this study was small, and the participants were recruited from a city where inhabitants tended to receive optimal medical care, potentially leading to a certain survey bias. In the future, we plan to recruit participants from different regions of the country to further verify our conclusions. Second, the participants might have some activities during ambulatory blood pressure monitoring, which may affect the accuracy of the results and lead to a certain measurement bias. It is best to repeat ambulatory blood pressure monitoring in the future to ensure the accuracy of the results.

## 6. Conclusion

MH is a common state of hypertension. We found that the level and variability of SBP over the course of 24 hours and specifically during the daytime and nighttime in people with MH were higher than those in people with normotension or controlled hypertension. In addition, those indexes in people with MH were similar to people with SH. These findings may help to explain why people with MH have target organ damages that are similar to people with SH. However, it is often difficult to identify MH patients because of normal blood pressure in the clinic, which can lead to a relatively poor prognosis when finally diagnosed. Therefore, it is important to pay much attention to developing strategies to increase the clinical detection rate of MH. Screening, diagnostic, and treatment strategies need to be further explored. The results of this study suggest future studies to explore whether reducing the SBP level and variability in MH patients can improve clinical outcomes.

The article "Analysis of Systolic Blood Pressure Level and Short-Term Variability in Masked Hypertension" was retracted in 2023. Reasons: signs of a paper mill; suspected computer-generated content; unreliable results or conclusions; concerns about the data.

## Figures and Tables

**Figure 1:** A flow chart of the current study.

**Figure 2:** Comparison of systolic blood pressure parameters of ambulatory blood pressure monitoring in the four groups. (a) 24 h systolic blood pressure, (b) daytime systolic blood pressure, (c) nighttime systolic blood pressure, (d) 24 h systolic blood pressure load, (e) daytime systolic blood pressure load, (f) nighttime systolic blood pressure load, (g) 24 h systolic blood pressure standard deviation, (h) daytime systolic blood pressure standard deviation, (i) nighttime systolic blood pressure standard deviation, (j) 24 h systolic blood pressure coefficient of variation, (k) daytime systolic blood pressure coefficient of variation, (l) nighttime systolic blood pressure coefficient of variation, and (m) nocturnal systolic blood pressure decline rate.

**Table 1:** Comparison of baseline data of the four groups.

	Normotension group (*n* = 62)	Controlled hypertension group (*n* = 78)	Masked hypertension group (*n* = 69)	Sustained hypertension group (*n* = 41)	*t*/*Z*/*χ*^2^	*P* value
Age (years)	63 (54, 68)		65 (55.8, 74)	63 (57, 71)	75 (60, 77)	10.924	**0.012**
Male gender, *n* (%)	44 (71.0)		59 (75.6)	37 (53.6)	26 (63.4)	8.778	**0.032**
BMI (kg/m^2^)	23.4 (21.6, 25.9)		25.1 (23.4, 26.7)	25.4 (23, 28.2)	25.5 (23.8, 28.3)	12.486	**0.006**
Never smoking, *n* (%)	31 (50.0)		49 (62.8)	39 (56.5)	29 (70.7)	5.412	0.144
Drinking, *n* (%)	15 (24.6)		13 (16.7)	19 (27.5)	8 (19.5)	5.677	0.460
Physical exercise, *n* (%)	55 (90.2)		61 (78.2)	53 (76.8)	33 (80.5)	4.538	0.209
Course of hypertension (years)	-		10 (3.8, 20)	5 (0, 18)	20 (10, 25.5)	123.735	**<0.001**
Number of antihypertension drugs, *n* (%)						94.635	**<0.001**
0	60 (96.8)		14 (17.9)	31 (44.9)	4 (9.8)		
1	2 (3.2)		23 (29.5)	15 (21.7)	16 (39.0)		
2	0		32 (41.0)	16 (23.2)	15 (36.6)		
3	0		9 (11.5)	6 (8.7)	4 (9.8)		
4	0		0	1 (1.4)	2 (4.9)		
Clinical history, *n* (%)							
Diabetes	13 (21.0)		32 (41.0)	42 (60.9)	18 (43.9)	21.435	**<0.001**
Hyperlipidemia	42 (67.7)		64 (82.1)	60 (87.0)	33 (80.5)	7.977	**0.046**
Chronic kidney disease	0		5 (6.4)	4 (5.8)	1 (2.4)	4.714	0.164
Hyperuricemia	18 (29.0)		13 (16.7)	8 (11.6)	7 (17.1)	7.001	0.072
Coronary heart disease	13 (21.0)		20 (25.6)	20 (29.0)	10 (24.4)	1.136	0.768
Sleep apnea syndrome	8 (13.1)		16 (20.5)	14 (20.3)	2 (4.9)	6.257	0.100
Laboratory parameters							
TG (mmol/L)	1.2 (0.8, 2)		1.5 (1.1, 2.1)	1.5 (1, 2.1)	1.2 (0.9, 1.6)	8.645	**0.034**
TC (mmol/L)	4.3 (3.7, 5)		4.1 (3.6, 4.5)	4.5 (3.7, 5)	4.1 (3.5, 5)	4.460	0.216
LDL-C (mmol/L)	2.5 (1.8, 3.1)		2.2 (1.8, 2.7)	2.7 (1.8, 3.1)	2.4 (1.8, 2.8)	4.945	0.176
HDL-C (mmol/L)	1.1 (0.9, 1.4)		1 (0.9, 1.2)	1 (0.9, 1.4)	1.1 (0.9, 1.3)	3.927	0.269
FBG (mmol/L)	5.1 (4.8, 5.7)		5.4 (4.9, 6.1)	5.7 (5.2, 7)	5.4 (4.9, 6.4)	13.950	**0.003**
HbA1c (%)	5.7 (5.5, 6.3)		6.1 (5.7, 6.6)	6.3 (5.9, 7)	6.1 (5.9, 6.8)	21.847	**<0.001**

Bold values represent the significant difference.

The article "Analysis of Systolic Blood Pressure Level and Short-Term Variability in Masked Hypertension" was retracted in 2023. Reasons: signs of a paper mill; suspected computer-generated content; unreliable results or conclusions; concerns about the data.

## Data Availability

No data were used to support this study.
